# Senotherapy Protects against Cisplatin-Induced Ovarian Injury by Removing Senescent Cells and Alleviating DNA Damage

**DOI:** 10.1155/2022/9144644

**Published:** 2022-06-03

**Authors:** Dingfu Du, Xianan Tang, Yufeng Li, Yueyue Gao, Runhua Chen, Qian Chen, Jingyi Wen, Tong Wu, Yan Zhang, Huan Lu, Jinjin Zhang, Shixuan Wang

**Affiliations:** ^1^Department of Obstetrics and Gynecology, Tongji Hospital, Tongji Medical College, Huazhong University of Science and Technology, Wuhan, Hubei 430030, China; ^2^Sun Yat-sen University Cancer Center, State Key Laboratory of Oncology in South China, Collaborative Innovation Center of Cancer Medicine, Guangzhou, Guangdong 510000, China; ^3^National Clinical Research Center for Obstetrical and Gynecological Diseases, Wuhan, Hubei 430030, China; ^4^Key Laboratory of Cancer Invasion and Metastasis, Ministry of Education, Wuhan, Hubei 430030, China; ^5^Department of Head and Neck Surgery, Sun Yat-sen University Cancer Center, Guangzhou, Guangdong 510000, China; ^6^Reproductive Medicine Center, Tongji Hospital, Tongji Medical College, Huazhong University of Science and Technology, Wuhan, Hubei 430030, China

## Abstract

Ovarian damage induced by platinum-based chemotherapy seriously affects young women with cancer, manifesting as infertility, early menopause, and premature ovarian insufficiency. However, effective prevention strategies for such damage are lacking. Senescent cells may be induced by chemotherapeutic agents. We hypothesized that cisplatin can lead to senescence in ovarian cells during the therapeutic process, and senolytic drugs can protect animals against cisplatin-induced ovarian injury. Here, we demonstrated the existence of senescent cells in cisplatin-treated ovaries, identified the senescence-associated secretory phenotype, and observed significant improvement of ovarian function by treatment with metformin or dasatinib and quercetin (DQ) independently or in combination. These senotherapies improved both oocyte quality and fertility, increased the ovarian reserve, and enhanced hormone secretion in cisplatin-exposed mice. Additionally, attenuated fibrosis, reorganized subcellular structure, and mitigated DNA damage were observed in the ovaries of senotherapeutic mice. Moreover, RNA sequencing analysis revealed upregulation of the proliferation-related genes *Ki*, *Prrx2*, *Sfrp4*, and *Megfl0*; and the antioxidative gene *H2-Q10* after metformin plus DQ treatment. Gene ontology analysis further revealed that combining senotherapies enhanced ovarian cell differentiation, development, and communication. In this study, we demonstrated that metformin plus DQ recovered ovarian function to a greater extent compared to metformin or DQ independently, with more follicular reserve, increased pups per litter, and reduced DNA damage. Collectively, our work indicates that senotherapies might prevent cisplatin-induced ovarian injury by removing senescent cells and reducing DNA damage, which represent a promising therapeutic avenue to prevent chemotherapy-induced ovarian damage.

## 1. Introduction

With the rapid development of modern medicine, multiple cancers have been rapidly, accurately diagnosed and treated in the early stage. Thus, the survival time of cancer patients has been significantly prolonged [1]. Acute lymphoblastic leukemia and breast cancer are the most common malignancies among female populations of adolescent and reproductive ages, respectively. The 10-year survival rate of the former exceeds 80%, and the five-year survival rate of the latter has reached 70% [2, 3]. Since a variety of tumor incidences gradually approach the young population, the quality of life of cancer survivors has become a growing problem needing urgently to be solved.

At present, chemotherapy remains the most prevalent treatment for cancer. Cisplatin is a first-line drug extensively used for various solid tumors, such as acute lymphoblastic leukemia, breast cancer, and cervical cancer, and it has been widely studied for its multisystem side effects [4]. Female gonads are particularly sensitive to cisplatin. Evidence suggests that the principal manifestation of cisplatin-induced ovarian damage is a loss of the healthy ovarian reserve and female fertility, frequently accompanied by increased atretic follicles [5]. The precise mechanisms underlying this drug's ovarian toxicity involve irreversible DNA damage, overloaded oxidative stress, and uncontrolled apoptosis activation [5–7]. Fertility-preservation strategies, such as ovarian tissue cryopreservation, embryo cryopreservation, stem cell transplantation, and oocyte donation, might benefit a proportion of tumor survivors. However, practical problems, such as safety and ethical issues, have restricted their wide use [8, 9]. Currently, no better method exists for recovering cisplatin-induced ovarian damage, and effective interventions can only be carried out if the involved mechanisms are uncovered.

Cellular senescence can be triggered by various stress stimuli and is characterized by permanent cell cycle arrest, macromolecular damage, deregulated cell metabolism, and a particular senescence-associated secretory phenotype (SASP), which can be detected by short, dysfunctional telomeres, persistent DNA damage response (DDR), P16^link4a^ expression, *β*-galactoside (*β*-gal) staining, and SASP [10, 11]. Cellular senescence inevitably occurs in normal aging tissues, and lingering senescent cells impair tissue homeostasis, further rendering aged tissues dysfunctional and vulnerable to stress [12]. Based on this theory, animal studies are in progress to evaluate the benefits of senotherapies in age-associated disorder prevention and healthy lifespan extension, and several approaches have been offered either involving the removal of senescent cells (such as ﻿dasatinib plus ﻿quercetin [DQ]) or the inhibition of SASP (such as metformin) secretions [13]. Recent evidence has reported that ﻿ DQ induces selective apoptosis of senescent cells (SNCs), preserves organ function, prevents age-related pathologies, and increases lifespan [14–16]. Metformin, a traditional ﻿antihyperglycemic agent, was recently identified to possess a senomorphic effect and the potential to fight against age-related diseases [17–19]. In addition to natural aging, studies into genotoxic agents, such as cisplatin, cyclophosphamide, and doxorubicin, have acknowledged their senescence-promoting effects [10, 20–22]. Surveys of cisplatin have shown that this chemotherapy could induce SNCs in normal tissues such as the kidneys and neurons, which are involved in the pathogenesis of acute kidney injury and peripheral neuropathy [23, 24]. To date, few attempts have been made to identify whether SNCs exist in cisplatin-exposed ovaries and whether senotherapies could protect against cisplatin-induced ovarian damage.

In our present research, we hypothesized that cisplatin might induce ovarian cell senescence and senotherapies may effectively restore ovarian reserve and function. Our study confirmed that DNA damage and SNCs were involved in the ovarian damage induced by cisplatin. Treatment with metformin or ﻿DQ alone or both in combination alleviated cisplatin-induced ovarian dysfunction by removing SNCs, inhibiting SASP secretion and blocking apoptosis. Our work uncovers a novel mechanism for cisplatin-induced ovarian damage and reveals that senotherapies targeting senescent cells may be a potential fertility-preservation avenue for female cancer patients.

## 2. Methods and Materials

### 2.1. In Vitro Primary Granulosa Cells (GCs) Culture and Drug Administration

Ovaries were isolated from euthanized 3-week-old female C57BL/6 mice and punctured thoroughly to release GCs. The harvested GCs were centrifuged at 800 revolutions per minute (rpm) for 5.5 minutes, incubated in DMEM/F12 (12400-024; Gibco Laboratories, Gaithersburg, MD, USA) culture medium, and then divided into 4 groups. The GCs of the blank control group (NC group) were treated with DMEM/F12 growth medium without any other treatment. For the cisplatin group (Cis group), cisplatin plus metformin group (Cis+M group), and cisplatin plus DQ group (Cis+DQ group), cisplatin (30 *μ*mol/L) was added to the medium after GC attachment. Following 24 hours, the whole medium of each group was replaced. GCs in the NC group and Cis group were cultured in DMEM/F12 growth medium for another 24 hours, and the other two groups were treated with metformin (5 mmol/L) or D+Q (D: 1 nmol/L; Q: 20 *μ*mol/L) for another 24 hours.

### 2.2. Cell Culture Medium Cytokine Detection

After drug administration, the cell culture medium of the NC group and Cis group was collected. The cytokines accumulated in culture medium after different medications were determined using a Luminex mouse 23 cytokine array (Wayen Biotechnologies, Shanghai, China).

### 2.3. Animal Care and Drug Administration

One hundred sex-mature 6-week-old C57BL/6 female mice were provided by the Tongji Hospital Experimental Animal Center, which is affiliated with the Tongji Medical College of Huazhong University. Animals were acclimated to the environment for one week before drug administration on an alternating 12-hour light/dark cycle with free access to food and water. Then, 20 mice were administered dasatinib (5 mg/kg) and quercetin (50 mg/kg) intragastrically 2 times weekly for 4 weeks and/or received metformin-containing water (2 mg/mL) or pure water over a period of 4 weeks (Cis+DQ, Cis+M, cisplatin plus metformin, and DQ [Cis+M+DQ] groups, 20 mice per group, 60 mice in total). One week after senotherapy administration, the aforementioned 60 mice were simultaneously subjected to intraperitoneal injection with 2.5 mg/kg of cisplatin 3 times weekly for the next 3 weeks. Another 20 mice received saline or cisplatin injection only at 7 weeks of age (NC and Cis groups, 20 mice per group, 40 mice in total). All animal operations were performed in compliance with the guide approved by the ethics committee of Tongji Hospital, Tongji Medical College, Huazhong University of Science and Technology, in the People's Republic of China.

### 2.4. Senescence-Associated- (SA-) *β*-Gal Staining

SA-*β*-gal staining of GCs or frozen ovarian slices was conducted according to the product manual. In brief, for GCs, samples were prewashed with phosphate-buffered saline and then fixed with the fixative solution provided in the Senescence *β*-Galactosidase Staining Kit (C0602; Beyotime Biotechnology, Haimen, China). For frozen ovarian sections, ovarian slices were rewarmed first and then processed for the staining step.

### 2.5. Sirius red Staining

A series of representative ovarian sections in different medication groups were chosen to identify the fibrosis level using Sirius red staining. Initially, we dewaxed and hydrated the ovarian slices and processed them with 10-minute celestine blue staining. After 3 washes with ddH_2_O, the ovarian sections were subjected to Sirius red solution for 30 minutes. Following another round of dehydration, we mounted ovarian slices with neutral resins for subsequent imaging and quantitative analysis.

### 2.6. Immunoblot and Quantitative Analyses

In brief, total ovarian proteins or proteins from cell lysates were extracted and separated by 10% sodium dodecyl sulphate–polyacrylamide gel electrophoresis (SDS-PAGE) gel or 12% SDS–PAGE gel according to the molecular weight of the proteins to be measured. Targeted proteins were subsequently transferred to polyvinylidene fluoride membranes and blocked with rapid blocking buffer for 30 minutes. After 3 washes with Tris-Buffered Saline and Tween 20 (TBST), targeted proteins were incubated with specific primary antibodies against nuclear factor kappa-light-chain-enhancer of activated B-cells (NF-*κ*B) (Cat# 10745-1-AP, 1 : 1000; Proteintech, Rosemont, IL, USA), P16^link4a^ (Cat# 10883-1-AP, 1 : 500; Proteintech, Rosemont, IL, USA), P21﻿^WAF1/Cip1^ (Cat# A1438, 1 : 1000; ABclonal Technology, Woburn, MA, USA), interleukin (IL)-6 (Cat# A0286, 1 : 1000; ABclonal Technology, Woburn, MA, USA), IL-1*β* (Cat# A19635, 1 : 500; ABclonal Technology, Woburn, MA, USA), proliferating cell nuclear antigen (PCNA) (Cat# sc-56, 1 : 1000; Santa Cruz Biotechnology, Dallas, TX, USA), heme oxygenase (HO)-1 (Cat# 10701-1-AP, 1 : 1000; ABclonal Technology, Woburn, MA, USA), and superoxide dismutase (SOD)2 (Cat# Ag21388; ABclonal Technology, Woburn, MA, USA) diluted in TBST overnight in a 4°C refrigerator. After 30 minutes of rewarming, target blots were washed with TBST 3 times and incubated with appropriate secondary antibodies for 1 hour the next day. Ultimately, blots were imaged using the chemiluminescence method after 3 washes.

### 2.7. Immunohistochemistry (IHC) and Immunofluorescence (IF) Staining

Three representative sections of ovaries in distinct groups were selected for IHC and IF analyses. The former was used to detect the localization and quantitative expressions of ovarian P16^link4a^, P21^﻿WAF1/Cip1^, IL-6, and 8-hydroxy-2 deoxyguanosine (8-OHdG) (Cat# sc-393871, 1 : 100; Santa Cruz Biotechnology, Dallas, TX, USA), and the latter was applied to identify zona pellucida protein 3 (ZP3) protein expression (ab70384, 1 : 100; Abcam, Cambridge, UK). IHC and IF were performed using routine protocols as previously described [25].

### 2.8. Terminal Deoxynucleotidyl Transferase dUTP Nick End Labeling (TUNEL) Cell Apoptosis Analysis and 5-Ethynyl-2′-Deoxyuridine (EdU) Cell Proliferation Analysis

Ovarian sections were first dewaxed and hydrated, and then we performed staining steps according to the manuals of the Colorimetric TUNEL Apoptosis Assay Kit (C1098; Beyotime Biotechnology, Haimen, China) and BeyoClick™ EdU Cell Proliferation Kit with Alexa Fluor 488 (C0071S; Beyotime Biotechnology, Haimen, China).

### 2.9. Transmission Electron Microscope

Three ovaries per group were preserved in electron microscope preservation solution (G1102; Servicebio, Wuhan, China). Transmission electron microscopy images of each ovary sample were taken by ServiceBio (Wuhan, China).

### 2.10. Estrous Cycle Analysis

Vaginal smears of all animals were sampled at 9:00 a.m. for 15 consecutive days from the day drug administration was finished. Vaginal secretions were collected with saline and then spread on slides, followed by hematoxylin and eosin (HE) staining after air drying. Then, the stage of the estrous cycle was determined by cytology by 2 people separately under a microscope.

### 2.11. Follicle Counting

Five ovaries from distinct individuals in each group were obtained for follicle counting. Dissected ovaries were preserved in 4% paraformaldehyde and then cut into 5 *μ*m pieces. Follicles at different levels were counted by 2 people separately. The detailed procedures were performed as previously described [26].

### 2.12. Serum Anti-Müllerian Hormone (AMH) and Estradiol (E_2_) Determination

Nonhemolytic blood samples of female mice were collected before sacrifice. Levels of serum AMH and E_2_ were determined using the Mouse AMH ELISA Kit and Mouse E_2_ ELISA Kit according to the manufacturer's instructions (CSB-E13156 m and CSB-E05109 m; Cusabio Technology LLC, Houston, TX, USA).

### 2.13. Mating Test

Five female mice in each group were randomly selected for the mating test. The mating test began once the drug administration ended. In brief, 10 days were designated as a mating cycle, and 2 female mice with 1 male mouse were arranged in one cage for mating. We tested the vaginal plugs every morning at 9:00 a.m. to evaluate for a pregnant outcome. The pregnant mice were then allocated to an independent cage, and their pup conditions were recorded. Ten days later, nonpregnant mice were marked and separated from male mice. After the first round parturition ended, another mating cycle was repeated. The duration of the mating test was 6 months in total.

### 2.14. Statistical Analysis

Statistical analyses were conducted using the SPSS 26.0 software (IBM Corporation, Armonk, NY, USA). Group differences of continuous variables were calculated using one-way analysis of variance (nonparametric tests). Group differences in regular cycle numbers were analyzed using chi-squared analysis. *p* < 0.05 was considered statistically significant.

## 3. Results

### 3.1. Confirmation of Senescent Ovarian Cells Induced by Cisplatin and Alleviated by Senotherapies

To determine whether cisplatin could induce ovarian cell senescence, we exposed ovarian GCs of female mice to cisplatin in vitro. The flowchart of in vitro experiment is shown in Figure 1(a). We first screened senescent stress via SA-*β*-gal staining. As shown in Figures 1(b) and 1(c), SA-*β*-gal–positive staining was remarkably increased in cisplatin-treated GCs relative to the control group (*p* < 0.05). To better investigate the secretory phenotype, cell culture medium following cisplatin administration was collected and determined using a Luminex mouse 23 cytokine array (Wayen Biotechnologies, Shanghai, China). Compared to the control, IL-6 obviously accumulated in the Cis group culture medium (*p* < 0.05, Figure 1(d)). Other inflammatory cytokines, such as granulocyte colony-stimulating factor (G-CSF) and IL-12 (P40), showed an upward trend following cisplatin administration without statistical significance (Figures 1(e) and 1(f)). The above results indicated that cisplatin might induce granular cell senescence.

To further explore whether senotherapies metformin and/or DQ may alleviate the senescence stress caused by cisplatin in vitro, we undertook western blot analysis of senescence-related markers. Quantitative analysis of senescence-related proteins in each group revealed significant upregulation of the senescence marker P21﻿^WAF1/Cip1^ and activation of ﻿NF-*κ*B in cisplatin-exposed GCs lysates (*p* < 0.05, Figures 1(g)–1(l)); however, another senescence effector, P16^link4a^, only shows an increased tendency (Figure 1(k)). Conversely, DQ administration led to an obvious downregulation of the senescence markers P21﻿^WAF1/Cip1^ and P16^link4a^ (*p* < 0.05) (Figures 1(k) and 1(l)), and metformin treatment only reduced P21﻿^WAF1/Cip1^ expression (*p* < 0.05, Figure 1(l)), suggesting metformin had a less profound senolytic effect than DQ. Western blot analysis of the SASP markers indicated that metformin excessively prohibited inflammatory cytokine secretion, and IL-6 and IL-1*β* in cell lysates were highly enriched after metformin treatment (*p* < 0.05, Figures 1(h) and 1(i)). Collectively, these results indicated that metformin and DQ variously attenuated the cisplatin-induced ovarian cell senescence burden in vitro. Of note, DQ exhibited a prominent senescent GC elimination capacity, and metformin probably acted via effective blockage of SASP secretion.

### 3.2. Removal of Senescent Cells by Metformin or DQ Alone or Both in Combination following Cisplatin Chemotherapy

To further reveal whether metformin and/or DQ intervention could mitigate senescent stress in vivo, we established a cisplatin-induced ovarian damage animal model to assess SNCs after the aforementioned medication. The flowchart of the animal experiment is shown in Figure 2(a). SA-*β*-gal staining of ovarian sections showed a trend consistent with that of the in vitro experiments. In particular, enlarged SA-*β*-gal–positive staining of mouse ovaries was recorded after cisplatin administration, and metformin and/or DQ invention resulted in various shrinkages of the SA-*β*-gal–positive staining area in the ovaries (*p* < 0.05, Figures 2(b) and 2(d)). Likewise, we determined senescence-associated markers in ovaries post cisplatin exposure. IHC results revealed remarkably increased positive expressions of P16^link4a^, P21^﻿WAF1/Cip1^, and IL-6 in cisplatin-treated ovaries, suggesting that senescence stress was also induced by cisplatin in vivo (Figure 2(c)). Alone or combined treatment with metformin and DQ significantly inhibited the expression of P16^link4a^, P21^﻿WAF1/Cip1^, and IL-6 (Figure 2(c)). Quantitative analysis of integral optical density (IOD) indicated that metformin plus DQ treatment removed the maximum senescence signal (*p* < 0.05, Figures 2(e)–2(g)). In summary, these data validated that senescent cells do exist in cisplatin-treated mouse ovaries, and ovarian senescent stress induced by cisplatin can be effectively removed by metformin and/or DQ treatment in vivo. In particular, metformin plus DQ treatment maximally eliminated the senescent burden in the cisplatin-exposed ovarian setting.

### 3.3. Reversal of Ovarian Function by Metformin or DQ Alone or Both in Combination against Cisplatin-Induced Damage

To further uncover whether metformin and/or DQ senotherapies protect ovaries from cisplatin-induced ovarian dysfunction, we undertook ovarian fibrosis evaluation, ovarian follicle counting, and estrous cycle and serum hormone determination in each group. Series of ovarian Sirius red staining indicated obvious fibrosis in cisplatin-treated ovaries, which was significantly alleviated following metformin and/or DQ administration (*p* < 0.05, Figures 3(a) and 3(h)). Ovarian follicle counting directly reflected the ovarian reserve. In this study, primordial follicles and growing follicles were largely reduced in cisplatin-treated ovaries, and atretic follicles were significantly elevated (*p* < 0.05, Figure 3(c)). However, metformin and/or DQ treatment restored the growth and development of ovarian follicles (Figure 3(c)). Notably, combination administration of both maximally preserved ovarian reserve and prohibited follicle atresia caused by cisplatin (*p* < 0.05, Figure 3(c)).

The estrous cycle is thought to be a reflection of ovarian endocrine function. We next assessed irregular estrous cycle frequencies in each group. Remarkably, cisplatin treatment disturbed estrous cycles in mice, as the percentage of irregular estrous cycles was up to 78.9% (*p* < 0.05, Figure 3(d)), with irregular estrous cycle rates of 50%, 47.4%, and 38.9% in the Cis+M group, Cis+DQ group, and Cis+M+DQ group, respectively (*p* < 0.05, Figure 3(d)). Moreover, the ovarian index was obviously reduced in cisplatin-treated mice, whereas senotherapies (Cis+M, Cis+DQ, and Cis+M+DQ) led to a significant recovery (*p* < 0.05, Figure 3(e)). To evaluate murine ovarian endocrine function post medication accurately, we measured the serum concentrations of E_2_ and AMH. Consistent with previous reports, serum E_2_ levels dramatically decreased after cisplatin exposure (*p* < 0.05, Figure 3(g)). Combination treatment with metformin and DQ reversed the decline in serum E_2_ levels in mice; however, no significant improvement in serum E_2_ levels was observed in the Cis+M and Cis+DQ groups (Figure 3(g)). Markedly decreased serum AMH (a predictive biological marker of ovarian reserve) in cisplatin-treated mice was also observed, while elevated serum AMH was recognized in the Cis+M, Cis+DQ, and Cis+M+DQ groups compared with cisplatin-exposed mice (*p* < 0.05, Figure 3(f)). Similarly, serum AMH was significantly improved in the Cis+M+DQ group, albeit remaining barely different from the NC group mice (Figure 3(f)). Taken together, cisplatin severely impaired mouse ovarian health reserve and function, and senotherapies metformin and/or DQ effectively reversed the injury.

### 3.4. Preservation of Fertility and Reshaping of Ovarian Subcellular Structure by Metformin or DQ Pretreatment

To identify whether metformin and/or DQ mitigates cisplatin-induced reproductive dysfunction and oocyte impairment, we performed a mating test. The general status of pups in each medication group is shown in Figure 4(a). The successful pregnancy rate in cisplatin-treated mice was significantly lower than that in the NC group, which was recovered in the Cis+M, Cis+DQ, and Cis+M+DQ groups (Figure 4(b)). Meanwhile, the pup mortality rate of cisplatin-treated mice increased compared to that of NC mice, and administration of metformin or DQ alone or both in combination seemed to decrease pup mortality (Figure 4(c)). Additionally, the average pup number per litter in the Cis+M, Cis+DQ, and Cis+M+DQ groups mice was significantly greater than that in cisplatin-treated mice (*p* < 0.05, Figure 4(d)). Notably, the number of pups per litter was indistinguishable between the combo medication group and the NC group (Figure 4(d)).

Healthy follicles constitute the elementary units of female ovaries. GCs serve as vital compartments of the follicle unit, suffering severe damage during cisplatin exposure. To disclose the influence of SNCs on granular subcellular structure, transmission electron microscopy was conducted to record subcellular morphologic alternations of GCs in distinct groups (Figure 4(e)). The majority of GCs were well aligned with integrated nuclear membranes, visible nucleoli, and evenly distributed chromatin in the NC group. Abundant good shapes of the subcellular organelles were captured by cameras, including oval and complete mitochondria with clear cristae and plentiful and enlarged reticulum with ribosome attachments, suggestive of functional protein synthesis. Conversely, the GCs in the Cis group showed a morphology of severely damaged subcellular ultrastructure, characterized by expansive perinuclear space, inhomogeneous distributed chromatin, increased heterochromatin, and even emergence of plasmarrhexis. The functional organelles also suffered from cisplatin exposure. We noticed that mitochondria were dissolved into vacuoles accompanied by discrete cristae, and the endoplasmic reticulum was swollen and even ruptured in cisplatin-exposed GCs. However, metformin, DQ, and metformin plus DQ combined treatment attenuated the subcellular deterioration caused by cisplatin. Compared to cisplatin-treated GCs, the distribution of chromatin was relatively uniform, along with rare heterochromatin, clear nuclear membrane, and limited perinuclear space after senotherapies. The subcellular organelles of the senotherapeutic groups appeared to have a good outline under transmission electron microscopy. The above results illustrated that cisplatin exerted a robust toxic effect on granular subcellular structure, and metformin, DQ, and metformin plus DQ in combination may counteract the subcellular toxic effect caused by cisplatin.

Essentially, oocyte quality is the primary determinant of female fertility and reproductive health. Previous literature has reported the direct impairment of oocytes caused by cisplatin [27]. Ovarian section ZP3 IF was further applied to assess oocyte quality via evaluation of zona pellucida conditions. Remarkably reduced healthy follicles but increased shrinking atretic follicles in cisplatin-treated ovaries were recorded via ZP3 staining. The administration of metformin and/or DQ was associated with an upregulation of normal ZP3 staining, indicating a restoration of oocyte quality following senotherapies (Figure 4(f)). These above results indicated that metformin and/or DQ administration reorganized the granular subcellular structure, preserved female mice fertility, and prohibited oocyte deterioration after cisplatin treatment.

### 3.5. Alleviation of Cisplatin-Induced Ovarian DNA Damage by Metformin or DQ Alone or Both in Combination

As reported, DDR is an important inducer of cellular senescence [28]. Previous studies have acknowledged DNA damage in other tissues caused by cisplatin and the emerging therapeutic effects of senolytics and senomorphics on organ dysfunction [13, 29]. Thus, we measured DNA damage levels via 8-OHdG IHC staining to identify the possible ovarian genotoxicity caused by cisplatin and the protective effects of senotherapeutic agents. Increased positive staining of 8-OHdG was observed in the Cis group, and western blot analysis revealed a significant decline in the antioxidative markers HO-1 and SOD2 in ovaries following cisplatin chemotherapy, indicating dramatic DNA oxidative injury and unmatched antioxidative capacity in cisplatin-treated ovaries (*p* < 0.05, Figures 5(a), 5(d), 5(g), and 5(h)). The above indexes were variously restored in ovaries treated by Cis+M, Cis+DQ, and Cis+M+DQ; among these, the combination treatment (Cis+M+DQ) ensured the largest elimination of ovarian DNA oxidative damage.

Additionally, the senolytics are suggested to take effect via the modulation of cell apoptosis [30]. To determine whether cisplatin-induced cell senescence affected ovarian cell viability, we performed TUNEL- and EdU-specific staining of ovarian sections to assess the status of cell apoptosis and proliferation in ovaries subjected to distinct treatments. Cisplatin chemotherapy resulted in severe apoptosis of ovarian cells (primarily GCs, small fraction of interstitial cells), while metformin, DQ, and metformin plus DQ co-administration treatment decreased the TUNEL staining (*p* < 0.05, Figures 5(b) and 5(e)). Positive EdU staining was almost invisible in cisplatin-treated ovaries; however, metformin, DQ, metformin+DQ combined treatment led to a notable recovery, as shown in Figures 5(c)–5(f). Statistical counting of the number of EdU–positive cells per square millimeter and quantitative analysis of PCNA proteins revealed cisplatin excessively activated the ovarian cell apoptosis, whereas metformin, DQ, and metformin plus DQ treatment reversed this process and restored ovarian cells proliferation to various degrees (*p* < 0.05, Figure 5(f)–5(h)). Notably, metformin plus DQ treatment exhibited the best cell protective capacity. In summary, metformin and/or DQ effectively protected ovaries from cisplatin-induced DNA damage.

### 3.6. Positive Regulation of Cell Development in Cisplatin-Induced Ovaries by Senotherapeutic Treatment

To explore the molecular events induced by senotherapies in cisplatin-treated ovaries, we employed transcriptome sequencing of ovaries in the different drug-administration groups. Venn diagrams show the number of differentially expressed genes (DEGs) between NC and Cis ovaries along with the rescued genes in different senotherapeutic groups (Figures 6(a) and 6(b)). Specifically, cisplatin exposure resulted in the downregulation of 73 genes in the ovaries, among which metformin, senolytic DQ, and metformin and DQ together rescued 1, 3, and 70 of them, respectively (Figure 6(b)). Thirty-five cisplatin-upregulated genes were modulated following senotherapies—in particular, metformin, senolytic DQ, and metformin and DQ together reset 13, 5, and 31 of them (Figure 6(a)). A heat map unveils the specific DEGs involved. In comparison to Cis-treated ovaries, cell proliferation-related DEGs, including *Ki*, *Prrx2*, *Sfrp4*, and *Megfl0*, and the antioxidative gene *H2-Q10*, were significantly upregulated in ovaries of the Cis+M+DQ group (Figure 6(f)). *Tnfrsf9* and another proliferation activator of endothelial cells, *Tnfrsf12a*, were modulated upwards following single metformin treatment (Figure 6(f)). Strikingly, senolytic DQ treatment downregulated the inflammatory-related gene *Cebpb* and the fibrosis-related gene *Loxl4* (Figure 6(f)). Moreover, DEGs between Cis-treated ovaries and different senotherapeutic groups were enriched in a series of gene ontology (GO) terms related to multiple cellular processes (Figures 6(c)–6(e)). Compared to the Cis group, senolytic DQ co-administration led to a significant enhancement of steroid hormone and lipid biosynthesis, and the genes associated with the cell-development process were also enriched after DQ treatment (Figure 6(d)). In addition, combination senotherapies (Cis+M+DQ group) facilitated cell differentiation, cell development, and cell signal communication (Figure 6(e)). The above comparative analysis of cisplatin and senotherapeutic DEGs in the ovaries supports the promotion effects of senotherapies on steroid hormone, cell proliferation, differentiation, and cell communication pathways, all of which are pathways that may contribute to fertility preservation in female cancer survivors.

## 4. Discussion

To date, chemotherapy is still the prevalent treatment for tumors and, among the available drugs, cisplatin is widely used in clinical practice. Cisplatin-induced ovarian damage primarily manifests as a loss of the healthy ovarian reserve and increased atretic follicles [5]. Currently, no effective medications are available to prevent such ovarian damage.

The underlying mechanisms of cisplatin-induced ovarian dysfunction involve irreversible DNA damage, overloaded oxidative stress, and uncontrolled apoptosis activation [5–7]. Recent evidence suggests that cisplatin not only leads to senescence of tumor cells but also affects peripheral nontumor renal and neuronal tissues [23, 24]. However, it remains unclear whether SNCs exist in cisplatin-exposed normal ovarian tissues. In our present study, we confirmed that cisplatin administration could induce ovarian cell senescence both in vitro and in vivo, and we further discovered that metformin and DQ treatment may improve cisplatin-injured ovarian function by removing senescent ovarian cells and reducing DNA damage.

DQ, a well-known senolytic, has shown a broad-spectrum senescent cell-killing effect. Emerging evidence suggests that senolytics targeting cell senescence may blaze a new trail for age-related diseases [13]. The cocktail of DQ has been reported to improve murine cardiac function and exercise capacity, thus delaying murine aging [30]. Metformin has been a widely used oral hypoglycemic medication for type 2 diabetes mellitus for five decades, and its nonglycemic benefits, including a prominent SASP elimination efficiency, have been consecutively identified in various in vitro and in vivo models [18, 19, 31]. In our present study, we confirmed the distinct senescence-removal effect and ovarian-preservation efficiency of metformin and/or DQ. Consistent with previous studies, metformin displayed a better SASP-inhibition ability, since western blot analysis showed a remarkable accumulation of SASP in cell lysates following metformin treatment. Importantly, dramatic downregulation of the senescent marker P21^﻿WAF1/Cip1^ was observed in Cis+DQ and Cis+M GCs, indicating a considerable senolytic capacity of DQ and metformin in the ovarian setting. Notably, in addition to SASP prohibition, metformin benefits ovaries by promoting *Sirt1* expression, preventing ovarian oxidative damage, ﻿reducing degenerating follicles and interstitial cells, and improving ovarian angiogenesis [32, 33]. Understandably, metformin plus DQ combination treatment produced a synergistic effect in cisplatin-exposed ovarian protection considering the complementary anti-aging targets of these 3 drugs. These data also supported the notion that the cell senescence burden is negatively correlated with ovarian health reserve and may probably work as a useful marker to predict female fecundity after cisplatin chemotherapy.

A hallmark of senescent cells is the secretion of SASPs or the senescence messaging secretome [10]. SASPs serve as mediators and spread senescence or senescence phenotypes in autocrine and paracrine fashions, thus interfere with cell viability and induce apoptosis [34]. We first set out to determine the SASPs secreted by senescent GCs following cisplatin exposure in vitro. A mouse cytokine array indicated significant elevation of inflammatory cytokine secretion in the cisplatin-exposed group; in particular, representative SASP IL-6 tripled over that in the NC group after cisplatin administration. The senomorphic agent metformin prominently alleviated SASP secretion after cisplatin exposure, since IL-6 and IL-1*β* were remarkably accumulated in cell lysates of Cis+M GCs compared to Cis-treated GCs. DQ showed a less profound influence on senescent granular SASP secretion, and IL-1*β* quantitative analysis showed an upwards tendency in cell lysates but reached no statistical significance compared to the Cis group. In addition, an in vivo animal experiment further demonstrated that cisplatin-induced ovarian cell senescence was not confined to GCs, since SA-*β*-gal staining and P16^link4a^- and P21^﻿WAF1/Cip1^-positive staining were also present in ovarian theca-interstitial cells. However, to determine whether theca-interstitial cell senescence is attributed to direct cisplatin damage or influenced by the SASP paracrine activity of GCs, further investigation is required.

In addition to the senescence removal of metformin and DQ discovered in our study, we surprisingly uncovered a metformin and/or DQ anti-DNA damage capacity in cisplatin-damaged ovaries. The antioxidative proteins SOD2 and HO-1 were significantly upregulated in the ovaries of the senotherapeutic groups, while subtle TUNEL staining and obvious EdU IF were noted in Cis+M, Cis+DQ, and Cis+M+DQ follicle units. Quantitative analysis of PCNA protein expression also revealed marked elevation after single or combined application of senotherapeutics. Transcriptome sequencing analysis further proved that the proportions of cisplatin-modulated genes could be rescued with single or combined senotherapies; of note, combination treatment rescued the largest proportion of genes. As expected, the heat map showed that cell proliferation-associated genes, such as *Ki*, *Prrx2*, *Sfrp4*, and *Megfl0*; and the antioxidative gene *H2-Q10* were remarkably enhanced in Cis+M+DQ ovaries. Except for senolytic efficiency, DQ probably exerted anti-inflammatory and antifibrosis effects since related genes were upregulated following DQ co-administration. GO enrichment analysis revealed that the biological processes enhanced after combination treatment were positive regulation of cell development, cell differentiation, and cell communication. Taken together, these data verified that senotherapies not only fight against cell senescence but also participate in multiple cellular processes and promote ovarian cell survival after chemotherapy in multiple ways.

Several limitations of our study should be declared here. First, we did not comprehensively detect all senescence-related markers in mouse ovarian tissue and GCs. Future studies are required to cover more SASPs and senescence markers. Second, we did not confirm our discovery in clinical samples, and associated experiments will be undertaken in the near future.

In summary, our present study demonstrated that cellular senescence is involved in cisplatin-induced ovarian dysfunction and clearance of senescent cells by independent or combined administration of metformin and/or DQ ameliorated cisplatin-induced ovarian dysfunction in mice. Metformin plus DQ therapy further attenuated cisplatin-induced DNA damage. Transcriptomic sequencing revealed that the proportions of cisplatin-altered genes were rescued and biological processes, such as cell differentiation, cell development, and cell signal communication, were significantly upregulated after combination treatment. Additionally, we discovered synergistic effects of metformin and DQ in cisplatin-induced ovarian failure. Our work provides a previously unreported mechanism for cisplatin-induced ovarian damage and reveals that senotherapies targeting senescent cells could partially reverse this damage and may represent a promising therapeutic avenue to prevent chemotherapy-induced fertility loss.

## 5. Conclusion

In conclusion, our work demonstrates that senotherapies might prevent cisplatin-induced ovarian injury by removing senescent cells and reducing DNA damage, which may serve as a promising therapeutic avenue to prevent chemotherapy-induced ovarian damage.

## Figures and Tables

**Figure 1:** Metformin and DQ independently reduced senescent granulosa cells and SASP caused by cisplatin in vitro. (a) Flowchart of primary GCs in vitro experiment. (b, c) Light microscopic images of SA-*β*-gal-stained GCs after cisplatin administration and quantitative analysis of SA-*β*-gal–positive GCs (*n* =3). Scar bars are marked on respective images. (d–f) Cytokines accumulated in cell culture medium of the NC and Cis groups. (g–l) The protein levels of senescence-associated markers and SASP were analyzed by western blotting (*n* =3). Results are presented using mean ± standard deviation values. ∗*p* < 0.05, ∗∗*p* < 0.01, ∗∗∗∗*p* < 0.0001.

**Figure 2:** Metformin or DQ alone or in combination with each other alleviated the senescent stress induced by cisplatin in vivo. (a) Flowchart of drug administration animal experiment. (b, c) Light microscopic images of SA-*β*-gal staining and P16^link4a^, P21^WAF1/Cip1^, and IL-6 IHC staining after different medications. Scar bars are marked on respective images (*n* =3). (d–g) Quantitative analysis of SA-*β*-gal–positive area and P16^link4a^-, P21^WAF1/Cip1^-, and IL-6-postive IOD (*n* =3). Results are presented using mean ± standard deviation values. ∗*p* < 0.05, ∗∗*p* < 0.01, ∗∗∗*p* < 0.001.

**Figure 3:** Metformin and DQ alone or with each other improved healthy ovarian reserve and function in cisplatin-treated mice. (a, h) Representative images of Sirius red stained ovaries and quantitative analysis of Sirius red positive area. Scar bars were marked on respective images (*n* =3). (b, c) HE staining of ovarian sections and quantitative counting of follicles at different levels (*n* =5). *Black arrow*: primordial follicle; *red arrow*: primary follicle, secondary follicle and antral follicle; *yellow arrow*: ﻿atretic follicle. (d) Regular and irregular estrous cycle percentage of different medication groups (*n* =6). (e) Mice ovarian index in different medication groups (*n* =10). (f, g) Serum AMH (*n* =8) and E_2_ (*n* =7) of following the administration of different drugs. Results are presented using mean ± standard deviation values. ∗*p* < 0.05, ∗∗*p* < 0.01, ∗∗∗*p* < 0.001.

**Figure 4:** Metformin or DQ alone or in combination with each other pretreatment reorganized the ovarian subcellular structure and preserved mice fertility. (a) General state of pups in different groups. (b–d) Successful pregnant rate, pup mortality rate, and pups per litter of the different drug-administration groups (*n* =5). (e) Transmission electron microscopy images revealed subcellular morphologies of different medication-treated ovaries (*n* =3). Red arrow: mitochondria; white arrow: endoplasmic reticulum (ER); blue arrow: vacuolated cytoplasm; N: nucleus of the GC. The low magnification was 3,000x and the high magnification (insets) was 10,000x. (f) Immunofluorescence of ZP3 in ovaries treated with different medication regimens (*n* =3). Results are presented using mean ± standard deviation values. ∗∗*p* < 0.01, ∗∗∗*p* < 0.001.

**Figure 5:** Metformin and DQ alleviate cisplatin-induced ovarian DNA damage. (a, d) Representative images of 8-OHdG immunohistochemical staining after different medications and quantitative analysis of 8-OHdG–positive expression based on IOD (*n* =3). (b, c, e, f) TUNEL and EdU fluorescence of ovarian sections after different medications and determination of TUNEL- and EdU-positive cell numbers (*n* =3). (g, h) Western blot analysis of SOD2, HO1, and PCNA protein expressions in ovaries treated with different medication regimens (*n* =3). Results are presented using mean ± standard deviation values. ∗∗*p* < 0.01, ∗∗∗*p* < 0.001.

**Figure 6:** Senotherapeutic treatment positively regulates cell development. (a, b) Venn diagrams of rescued DEGs. (a) The number of cisplatin enhanced genes downregulated by senotherapies. (b) The number of cisplatin downregulated genes recovered by senotherapies. (c–e) GO terms enriched based on DEGs between the Cis group and different senotherapeutic groups. (f) Heat map of DEGs ovaries treated with different medication regimens (*n* =3).

## Data Availability

The data that support the findings of this study are available from the corresponding author upon reasonable request.

## Abbreviations

DQ: Dasatinib and quercetin
SASP: Senescence-associated secretory phenotype
DDR: DNA damage response
*β*-gal: *β*-Galactoside
SNCs: Senescent cells
GCs: Granulosa cells
rpm: Revolutions per minute
SDS-PAGE: Sodium dodecyl sulphate–polyacrylamide gel electrophoresis
TBST: Tris-Buffered Saline and Tween 20
NF-*κ*B: Nuclear factor kappa-light-chain-enhancer of activated B-cells
IL: Interleukin
PCNA: Proliferating cell nuclear antigen
HO: Heme oxygenase
SOD: Superoxide dismutase
IHC: Immunohistochemistry
IF: Immunofluorescence
8-OHdG: 8-hydroxy-2 deoxyguanosine
ZP3: Zona pellucida protein 3
TUNEL: Terminal deoxynucleotidyl transferase dUTP nick end labeling
EdU: 5-Ethynyl-2′-deoxyuridine
HE: Hematoxylin and eosin
AMH: Anti-Müllerian hormone
E_2_: Estradiol
G-CSF: Granulocyte colony-stimulating factor
IOD: Integral optical density
DEG: Differentially expressed genes
GO: Gene ontology.

## References

[1] Sung H., Ferlay J., Siegel R. L. (2021). Global cancer statistics 2020: GLOBOCAN estimates of incidence and mortality worldwide for 36 cancers in 185 countries. *CA: a Cancer Journal for Clinicians*.

[2] Taylan E., Oktay K. H. (2017). Current state and controversies in fertility preservation in women with breast cancer. *World J Clin Oncol.*.

[3] Bhakta N., Liu Q., Ness K. K. (2017). The cumulative burden of surviving childhood cancer: an initial report from the St Jude Lifetime Cohort Study (SJLIFE). *Lancet*.

[4] Qi L., Luo Q., Zhang Y., Jia F., Zhao Y., Wang F. (2019). Advances in toxicological research of the anticancer drug cisplatin. *Chemical Research in Toxicology*.

[5] Spears N., Lopes F., Stefansdottir A. (2019). Ovarian damage from chemotherapy and current approaches to its protection. *Human Reproduction Update*.

[6] Nguyen Q. N., Zerafa N., Liew S. H. (2018). Loss of PUMA protects the ovarian reserve during DNA-damaging chemotherapy and preserves fertility. *Cell death & disease*.

[7] Ayres L. S., Berger M., de Oliveira Durli I. C. L. (2020). Kallikrein-kinin system and oxidative stress in cisplatin-induced ovarian toxicity. *Reproductive Toxicology*.

[8] Dolmans M. M., Manavella D. D. (2019). Recent advances in fertility preservation. *The Journal of Obstetrics and Gynaecology Research*.

[9] Harada M., Osuga Y. (2019). Fertility preservation for female cancer patients. *Fertility and sterility*.

[10] Gorgoulis V., Adams P. D., Alimonti A. (2019). Cellular senescence: defining a path forward. *Cell*.

[11] He S., Sharpless N. E. (2017). Senescence in health and disease. *Cell*.

[12] Childs B. G., Durik M., Baker D. J., Van Deursen J. M. (2015). Cellular senescence in aging and age-related disease: from mechanisms to therapy. *Nature Medicine*.

[13] Martel J., Ojcius D. M., Wu C. Y. (2020). Emerging use of senolytics and senomorphics against aging and chronic diseases. *Medicinal Research Reviews*.

[14] Ogrodnik M., Miwa S., Tchkonia T. (2017). Cellular senescence drives age-dependent hepatic steatosis. *Nature Communications*.

[15] Iske J., Seyda M., Heinbokel T. (2020). Senolytics prevent mt-DNA-induced inflammation and promote the survival of aged organs following transplantation. *Nature communications*.

[16] Xu M., Pirtskhalava T., Farr J. N. (2018). Senolytics improve physical function and increase lifespan in old age. *Nature medicine*.

[17] Chen D., Xia D., Pan Z. (2016). Metformin protects against apoptosis and senescence in nucleus pulposus cells and ameliorates disc degeneration in vivo. *Cell death & disease*.

[18] Hansel C., Barr S., Schemann A. V. (2021). Metformin protects against radiation-induced acute effects by limiting senescence of bronchial-epithelial cells. *International Journal of Molecular Sciences*.

[19] Hu Q., Peng J., Jiang L. (2020). Metformin as a senostatic drug enhances the anticancer efficacy of CDK4/6 inhibitor in head and neck squamous cell carcinoma. *Cell death & disease*.

[20] Palaniyappan A. (2009). Cyclophosphamide induces premature senescence in normal human fibroblasts by activating MAP kinases. *Biogerontology*.

[21] Meredith A. M., Dass C. R. (2016). Increasing role of the cancer chemotherapeutic doxorubicin in cellular metabolism. *The Journal of Pharmacy and Pharmacology*.

[22] Nacarelli T., Fukumoto T., Zundell J. A. (2020). NAMPT inhibition suppresses cancer stem-like cells associated with therapy-induced senescence in ovarian cancer. *Cancer Research*.

[23] Calls A., Torres-Espin A., Navarro X., Yuste V. J., Udina E., Bruna J. (2021). Cisplatin-induced peripheral neuropathy is associated with neuronal senescence-like response. *Neuro-Oncology*.

[24] Li C., Xie N., Li Y., Liu C., Hou F. F., Wang J. (2019). N-acetylcysteine ameliorates cisplatin-induced renal senescence and renal interstitial fibrosis through sirtuin1 activation and p53 deacetylation. *Free Radical Biology and Medicine*.

[25] Ma Y., Qi M., An Y. (2018). Autophagy controls mesenchymal stem cell properties and senescence during bone aging. *Aging Cell*.

[26] Zhang X.-m., Li L., Xu J.-j. (2013). Rapamycin preserves the follicle pool reserve and prolongs the ovarian lifespan of female rats via modulating mTOR activation and sirtuin expression. *Gene*.

[27] Nguyen Q. N., Zerafa N., Liew S. H., Findlay J. K., Hickey M., Hutt K. J. (2019). Cisplatin- and cyclophosphamide-induced primordial follicle depletion is caused by direct damage to oocytes. *Molecular Human Reproduction*.

[28] Van Deursen J. M. (2014). The role of senescent cells in ageing. *Nature Publishing Group*.

[29] Wang W. J., Chen X. M., Cai G. Y. (2021). Cellular senescence and the senescence-associated secretory phenotype: potential therapeutic targets for renal fibrosis. *Experimental Gerontology*.

[30] Zhu Y., Tchkonia T., Pirtskhalava T. (2015). The achilles’ heel of senescent cells: from transcriptome to senolytic drugs. *Aging Cell*.

[31] Noren Hooten N., Martin-Montalvo A., Dluzen D. F. (2016). Metformin-mediated increase in DICER1 regulates microRNA expression and cellular senescence. *Aging Cell*.

[32] Qin X., Du D., Chen Q. (2019). Metformin prevents murine ovarian aging. *Aging (Albany NY)*.

[33] Mahamed R. R., Maganhin C. C., Sasso G. R. S., de Jesus Simões M., Baracat M. C. P., Baracat E. C. (2018). Metformin improves ovarian follicle dynamics by reducing theca cell proliferation and CYP-17 expression in an androgenized rat model. *J Ovarian Res. Journal of Ovarian Research*.

[34] Acosta J. C., Banito A., Wuestefeld T. (2013). A complex secretory program orchestrated by the inflammasome controls paracrine senescence. *Nature Publishing Group*.

